RETRACTED

# Research on the inheritance and protection of folk art and culture from the perspective of network cultural governance

**DOI:** 10.1371/journal.pone.0246404

**Published:** 2021-02-11

**Authors:** Kai Zhou, Kainan Wang, Xinxin Lin

**Affiliations:** School of Cyber Security, Changchun University, Changchun, Jilin, China; University College London, UNITED KINGDOM

## Abstract

In the age of network, network culture is gestated, and the emergence of security issues makes the governance of network culture put on the agenda. In order to explore ways to protect and inherit folk art and culture, This article mainly uses the mathematical model established by the principal component analysis method and the multiple regression method to analyze the current folk arts such as the lack of professional talents and other problems faced by the current folk arts. From the perspective of network cultural governance Analyze the number of audiences, etc., and reflect the inadequacy of the inheritance and protection of folk art and culture through the model, Therefore, it is proposed to cultivate compound talents, build cultural brands, and build a "gatekeeper" defense line. While creating a clear cyberspace, it can achieve better protection and inheritance of folk art and culture.

## Introduction

Chinese folk art is a part of traditional Chinese culture. It comes from life, and after historical precipitation, it concentrates the group consciousness of the Chinese people in the form of art, and has a strong "symbolic" and "inheritance" to the common customs, values, behavioral patterns, and other elements of traditional Chinese culture [1].

As the fourth medium, the Internet is facing the current background of cultural globalization and Internet globalization. The inheritance and protection of our country’s folk culture and art has been strongly impacted, and many folk arts and cultures have been lost seriously. Therefore, it is necessary to inherit and protect folk art under the premise of network culture governance. With the continuous development of network technology, the security of network has been widely concerned. Xi Jinping believes that literature and art are the clarion call for the advancement of the times, which is the most representative style and feature and the most able to lead the ethos of an era [2]. Folk art, as an organic part of literature and art, how to safely use the Internet to spread and inherit it has become an important topic of network culture security from the perspective of Cyberspace Security.

In China, many scholars have conducted in-depth research on cultural governance and folk art communication. Li Yanzu [3] put forward the concept of original ecology and market state of folk art, and thought that the elite groups in the city made rational choice and transformation of folk art, making it a part of cultural industry in the city market. In today’s highly developed network, the choice of folk art has gradually expanded from the city to every corner with network, and the chosen group has also expanded to every netizen with the development of self media, and whether the choice is rational has become a question to be considered. Xia Zhaodong [4] believes that the deep-seated connotation of folk art has a trend of being eroded due to the influence of market conditions, and proposes measures to protect folk art based on new media. However, in today’s era of great changes in aesthetics, the market’s selection criteria for folk art need to be remeasured. In the competition between marginalized folk art and modern forms of expression, some folk arts that have not yet been mined out are difficult to emerge in the complex fragmented and visual impact forms. Self media based on interest point selection is hard to spread the aging and retro folk art forms on a large scale. Kirshenblatt-Gimblett [5] argues that cultural heritage, including folk art, needs to be re-evaluated, filtering out obsolete elements and giving them new life through exhibitions, including performances, in combination with new age ideas.

RETRACTED

In this paper, the spread of folk art will be analyzed from the perspective of cyberspace. Starting from the governance of network culture, the problems and challenges of folk art in cyberspace will be discussed, in order to provide professional suggestions for the spread and protection of folk art in the network.

## Problems

### 1. The audience of folk art and culture is not concentrated

The feudal society lasted for more than 2000 years in China. Folk art was born here and absorbed many nutrients from the soil of the feudal society, which included the living conditions of the folk people and their pursuit of official career in this historical stage, and described the contradictions among all classes in the feudal society. Although there are some elements of love and entertainment, the differences of aesthetic habits, cognitive level and social contradictions in the whole generation make folk art difficult to be accepted by the public and finally frustrated in communication. In addition, the self-sufficient individual economy and the way of thinking affect the development and inheritance of folk art. Under the constraints of transportation, communication and other technical means, it is difficult to form a whole of folk art in the decentralized state. Specific folk art representatives have unique stories behind them, and the basis for their spread is the interest and concern of the characteristic groups, which is unstable. At the same time, the constraints of communication between different regions make the information relatively blocked, so the same type of folk art produced in different regions lacks necessary information to coordinate and promote each other, therefore restricts the overall development.

RETRACTED

China has suffered a hundred years of aggression in modern times, and new things have spread from the West and the east to China. The attention of the people to new things has increased, while the folk art forms representing the local culture have declined in the competition with the new forms, and the underdetermined practitioners have changed careers, which has brought a heavy blow to the inheritance of folk art. In addition, people with lofty ideals have been studying abroad to find the way to save the country. The attention to folk art has been greatly reduced, and the feudal color of folk art is not accepted by the times. Folk art was in recession. Having experienced the changes of the times, some folk art masters’ persistence in art weakened. The determination of successors has become the last lifeline of folk art.

Today, the lack of audience for traditional folk art in the context of network cultural governance is mainly reflected in the lack of successors to folk art, the incomplete knowledge of folk art among the general public, and the generalized view that traditional folk art culture is outdated and backward. The folk art that has been passed down to this day is also slightly tired in the face of such a developed film and television industry, with the development of Internet mobile data, China’s traditional folk art and culture will also enter a new era of digital communication. The auditory and visual effects brought by the new forms of expression are more in line with the aesthetic needs of the masses today. Although the national society attaches great importance to traditional culture, the masses’ knowledge of folk art is limited and professionalism is strong, making it difficult for outsiders to mention it. Interests to appreciate, but professionals are relatively scattered, it is difficult to play an effective driving action to stimulate the masses to continue to pay attention to folk art, resulting in a scattered audience of folk art, the audience area is small, take shadow puppets as an example, when movies are popular in major theaters When broadcasts and new productions are endless, there are few shadow puppets, making this "predecessor of the movie" far less influential than the younger generation. In addition, folk art usually has a certain influence in various regions, but other regions lack recognition. Although the publicity methods are advanced, it is difficult to be attracted by folk art for a long time due to the fatigue of the masses. Folk art in each region is alone Development, hard support, no unified system.

RETRACTED

For a long time, people for the inheritance and development of folk art has a lot of misunderstanding, so much so that many people think that folk art is a simple, cheap, old, no technical content, and put folk art at a margin status, cannot get very good development, thus further ignore the DPP fresh and contemporary art. Moreover, many people believe that folk art is not innovative and cannot be combined with the contemporary background, which leads to insufficient protection, insufficient publicity and insufficient development of folk art, and further leads to insufficient understanding of traditional culture among the public, prejudice against it and rejection psychology, resulting in the loss of some folk art. Moreover, due to the rise of various modern information media and the increasing number of channels to obtain information, teenagers and young people cannot pay much attention to folk art and culture due to the huge amount of information they get. Therefore, more attention should be paid to the problem that the audiences of folk art and culture are not concentrated.

### 2. Lack of professional talents in folk art communication

On January 3, 2019, Luo Shugang, Minister of Culture, pointed out at the meeting of Directors of the National Department of Culture and Tourism in 2019 that "the total number of people covered by the training program for intangible cultural heritage inheritors in China has reached 71000." Although this marks the formation of new atmosphere and new pattern, it is far from the huge work of folk art protection and inheritance.

Talent cultivation needs to start from the basic team. Statistics from the website of the Ministry of Education of the people’s Republic of China on June 11, 2020 show that in 2019, the number of graduates of ordinary undergraduate schools in China was 3947157, including 59394 art graduates, accounting for 1.500%, 3623527 junior college graduates, including 51470 art graduates, accounting for 1.420%, and 632399 graduate students in China. There are 20758 Chinese art graduates, accounting for 3.282% (State Department of Education website statistics as of June 11, 2020: http://www.moe.gov.cn/s78/A03/moe_560/jytjsj_2019/qg/). In addition, Table 1 shows the specialty setting of arts in China.

**Table 1:** Art studies category major establishment.

Category	Bachelor’s degree program
Art Theory Class	Art History
Music and Dance Class	Musicology, Musical performance, Dancology, Nautch Composition and technical theory of composition, Choreography
Drama and Film-and-Television Class	Arts of broadcasting and anchoring, Radio and television editor, Film and TV Literature, Dramaturgy, filmology, Drama film director, Performance, Recording arts, Film and television photography and production (specialty), Art design of drama, film and television, Animation
Fine Arts Class	Fine arts, Drawing, Sculpture, Photography, Chinese painting (specialty), Calligraphy (specialty)
Design Science Class	Visual communication design, Environmental design, Product design, Clothing and costume design, Digital media art, Public art, Industrial art, Art design, Arts and technology (specialty)

Source: Ministry of Education of the People’s Republic of China Official Website. http://www.moe.gov.cn/srcsite/A08/moe_1034/s3882/201209/t20120918_143152.html.

RETRACTED

Among these 33 majors, four are related to drama and one is related to folk art, accounting for a relatively small proportion. Most art students are more inclined to new forms such as film and television, design, sculpture photography, etc., which makes the number of undergraduate students of folk art more unable to meet the needs of society.

Referring to the 2019 Alumni Association Ranking of China’s Art Universities, for example (data from the official website of the China Conservatory of Music (http://bkzs.ccmusic.edu.cn/)), the school enrolled 315 students in 2020, including 112 students in three directions of Chinese vocal music, Chinese opera and Chinese musical instrument performance under music performance, accounting for 34.46%. On the contrary, the enrollment prospectus of Jilin Conservatory of Art’s in 2020 shows the number of national music performers accounts for 25% of the total number. In drama and television major, broadcasting and hosting, aesthetic design, film and television are the main subjects. In addition, 75 people are enrolled in dance major to learn Chinese dance performance. 30 people are enrolled in opera performance to learn Beijing Opera and Jiju. Besides, there are a large number of animation, education, pop music and design majors.

From excellent universities to ordinary ones, the differences in resources, attention and sensitivity reflect that the cultivation awareness of folk art related talents needs to be further improved, and the problems of insufficient talents and uneven distribution are also prominent. A large number of excellent art colleges and universities and resources are concentrated in developed cities, so that students in small areas can ‘t get high-quality training resources.

RETRACTED

### 3. Insufficient participation in the dissemination of folk art and culture

For a long period of time, traditional folk art culture has been impacted by various entertainment cultures, and civil society’s interest in folk art has begun to decline. In the initial stage of the protection of folk art, the public had too little knowledge of folk art, and social forces did not have an accurate understanding of how to start this cause and what effect it needed to achieve. As a result, people’s social participation in folk art and cultural exchanges is not high enough. It is necessary to formulate corresponding policies at the national level to stimulate the development of this cause. During this period, the government’s “big package” approach made some people begin to pay attention to and embark on the process of protecting folk art, which promoted the development of this cause. Has its historical merits.

After the social cognition of folk art has reached a certain level, especially after cultural self-confidence is put forward, the public’s cognition of culture has improved. At this time, the government’s "take on all things" approach restricts the innovation and competition of social organizations and individuals. The cultural management department takes the completion of work tasks as its goal and lacks passion for the protection of folk art. This negative attitude is not conducive to the overall development of folk art. At the same time, some non-governmental organizations have no clear understanding of their own functions and have wrong working principles [6], which is not conducive to the improvement of their own thinking ability of cultural units and reasonably judge according to the actual situation, so that the protection of folk art loses its original meaning.

Universities, as research heights, play an important role in promoting the overall development of art. In this paper, the keyword "folk art" is searched from the China Knowledge Network (https://www.cnki.net/) to obtain the development trend of academic research in this research field, as shown in Fig 1. The tendency for this field to have a bottleneck in research, which makes it difficult to make huge breakthroughs.

**Fig 1:** Academic research trends in folk art universities. Source: https://www.cnki.net/.

In addition, with the gradual increase in the country and society’s demand for cultural industries, companies are facing difficulties in the development of cultural industries. Although companies have gradually shifted the direction of resource mining to traditional domestic culture in recent years, the results have been relatively small. Folk art is a tradition As an organic part of the culture, enterprises have less digging and paying attention to folk art. The community is the cell and unit of society. Although the influence of folk art is gradually increasing, the role of the community in the dissemination and display of folk art is really limited, and it has not or less as an effective organizational platform for communicating between folk art and community residents.

RETRACTED

As an important part of society, teenagers also play an important role in the participation of this cause. However, they make their voices according to their own interests in the form of individuals, families, school society, or students’ social practice can hardly catch widespread concern of the society. Therefore, there is a lack of leading organizations to integrate resources and form an overall plan to light the torch to protect folk art.

## Network communication of folk art

### 1. Network communication of folk art is the need of network development in the new era

Since China formally connected to the Internet in 1994, the network has gradually changed people’s daily life, caused people’s different degree of thinking in many fields, and deeply affected people’s production mode. But as the field of network penetration becomes wider and wider, the number of people using the Internet is increasing day by day. From 2010 to June 2019, the number of Internet users in China is shown in Fig 2.

**Fig 2:** Change histogram of internet users from 2010 to 2019. Source: CNNIC, China Industrial Research Institute(http://www.199it.com/archives/tag/cnnic).

As shown in Fig 1, in June 2019, the number of Internet users in China has reached 854.49 million, accounting for 61.237% of the total number of people (1395.38 million). Such a large number brings about the same complex problems, which attracted more and more attention of the society. After the definition of cyberspace as the fifth space, the attention to the security issues in cyberspace has been raised to a new height that can be demonstrated that Cyberspace Security has been set as a first-class discipline. In this environment, the network has brought new opportunities and challenges to the field of folk art. How to use the network to better inherit folk art and how to protect folk art more effectively has become an important topic in the cause of folk art protection.

Xi Jinping stressed that culture is an important force for the survival and development of the nation [2], culture plays a very important role in the process of realizing the Chinese dream. Based on the security challenges faced by the cultural transmission in cyberspace, the governance of cyber culture has been put on the agenda. Cultural governance is an important feature of contemporary China’s development and the pursuit of the goal of national governance [7], so how to transmit it safely and efficiently is widely discussed in the society. As a part of Chinese culture, the spread of folk art in cyberspace will be discussed under this framework.

RETRACTED

Taking the network dissemination of folk art and culture as an important part of the country and society’s vigorous development of cultural undertakings and cultural industries, on the one hand, is conducive to providing more colorful cultural food for the majority of netizens, and meeting people’s spiritual needs; On the one hand, it is conducive to making folk art more affect the lives of the majority of netizens, and balancing the appearance of Chinese and Western art content on online platforms. Therefore, vigorously spreading the value of folk art through the Internet is not only an inevitable channel for the development of folk art, but also a need for the development of the Internet in the new era.

### 2. The network communication of folk art is the need of its protection and inheritance

How to upload the folk art to the network space needs attention. On June 7, 2019, 5G began to be commercially used, marking that China has entered the 5G era. Looking back on the course from 2G to 5g, the expression form of information has gradually changed from text and picture to audio and video. The continuous update of virtual imaging technology, network and communication technology has provided a good choice for the download and preservation of folk art. With the support of Internet communication technology, the dissemination efficiency of folk art has been greatly improved, which not only allows traditional folk art and culture to subtly infiltrate people’s lives, but also allows the general public to participate in the creation of folk art, but only to adapt to the characteristics of the Internet era, the works made by the public in pursuit of individuality can win the attention of some netizens in the short term, but In the long term, the fragmentary works lack systematic planning and careful operation, so it is difficult to win the widespread and sustained attention of the public, and finally sink into the sea of information.

In cyberspace, how to protect and inherit folk art is not only the task of folk artists, but also the joint efforts of network experts and communication scholars. Due to the lack of necessary knowledge in management and technology, and the inability of management and technical personnel to accurately grasp the law of art, so caused divergence between them and can’t achieve the expected effect in the specific work. The cultivation of composite talents is an effective way to solve this problem.

RETRACTED

With the continuous updating of technology, a grim working environment has been brought. Many posts have been replaced by computers. With such a fast pace of life, people can only pay attention to their interest points through fragmentary time, and hard to spend a lot of time to understand folk art, or have a channel to contact the story behind folk art and form a whole cognition. All these have reduced the enthusiasm of the masses for folk art. Whether folk art can stand out from the mass fragmentary information, and does not violate the real connotation behind it depends on the wisdom of practitioners.

The arrival of COVID-19 in 2020 has caught the whole nation by surprise. People have to stay at home and cannot gather in large numbers. However, the spread and protection of folk art has gained new development. Based on a variety of short video APP, and the public, such as popular media, emerged a large number of folk art we are through the network to the spread of folk art, combined with epidemic and their own ability, creating a series of works, not only let more people know about folk art, at the same time increase one’s determination and confidence to overcome the outbreak, which makes the further spread of folk art, folk art has been more and more people are familiar with and get more people to love and support. Therefore, it is necessary to combine the protection and inheritance of folk art with the network in the current information age.

### 3. Strengthening the supervision of network communication of art is the need of constructing a clear network space

The Internet has promoted the pace of people’s pursuit of personalization, and people began to choose information based on their own interests. Although this has some progressive significance, it also brings some problems. In the flood of information, short video and network broadcast are the most popular form of expression at present, a large number of teenagers are obsessed with this enjoyment of visual and auditory pleasure, unable to extricate themselves; the popularity of network novels, a large number of meaningless, plagiarized essays has also won a large number of viewers, which influence the way of people’s thinking and easy to form for teenagers wrong values. Due to factors such as low threshold, large revenue and wide audience, network broadcast platform is not strictly supervised, and problems such as pornography, violence and infringement are very prominent, which cause extremely serious harm to the society and easily lead to the formation of a bad social atmosphere. With the development of self media, it is more convenient for the public to carry out the secondary dissemination of information in the network on a certain issue, which inevitably including false and misinterpretation in the massive information. In addition, the attraction of the game to the public can’t be ignored. The rapid rise of the game industry and huge industrial profits reflect the direction of the current public interest. These information occupy a large amount of time and energy of the public, and it is difficult to contact the real connotation of folk art, so that the public can not form a correct understanding, which has a great impact on the dissemination and inheritance of folk art.

RETRACTED

The network makes the information break through the limitation of space and spread quickly. A large number of high-quality art forms from abroad attract many people’s attention. These contents arouse the public’s fresh feeling and have a certain impact on the public about the ideological thought, which has a negative impact on the spread of folk art. Although art knows no borders, the supporting point behind art is the culture of various nationalities. For example, the prevalence of Hollywood blockbusters has influenced the domestic teenagers a lot. Under the competition with these cultural products processed by high technology, Chinese folk art is difficult to get attention. The short-term audience number is also gradually decreased, which makes folk art communication have difficulty in carrying out a cause.

Beautiful China not only requires ecological balance, but also cyberspace clear. In the environment of building a community of shared destiny, discordant voices that wrapped in the shell of art always appear to erode the cognition of the masses in our country. There are also some negative energies spread by lazy and ignorant people in the society through the network, which need the government to identify and eliminate with a more scientific regulatory system, and build a clear environment for our country’s cyberspace.

## Research design

On the basis of the study of art and culture, the heritage and protection of folk art and culture are studied based on the network cultural environment and modeled based on principal component analysis and multiple linear regression models. The data is from China Culture and Tourism Statistical Yearbook(2019) (https://data--cnki--net--shjd.naihes.cn/yearbook/Single/N2020050235), China Culture and Related Industries Statistical Yearbook(2019) (https://data--cnki--net--shjd.naihes.cn/yearbook/Single/N2020030069).

### 1. Model building

It combines two models—principal component analysis (PCA) and multiple linear regression (MLR) methods. Principal component analysis involves spatially downscaling high-dimensional data variables and constructing several composite indicator variables (i.e., principal components) that are linear combinations of known indicator variables, which are relatively few in number and retain as much information about the original indicator variables as possible.

RETRACTED

Multiple Linear Regression Model is a mathematical formula that expresses a quantitative relationship between two or more independent variables, corresponding to one of the dependent variables, under the condition that the data of several indicator variables are linearly correlated.

#### Data downscaling

Sequentially find a set of mutually orthogonal axes from the space where the original indicator variable data are located, and ignore the remaining axes. First, mean and variance are computed for the sample, see Eqs (1) and (2):

$$\bar{X}=\frac{1}{n}\overset{n}{\underset{i=1}{\sum }}X_{i}$$ (1)

$$S^{2}=\frac{1}{n-1}\sum_{i=1}^{n}{\left(X_{i}-\bar{X}\right)}^{2}$$ (2)

Where $\bar{X}$ is the mean of the variable, *S*^2^ is the variance of the variable, n is the number of samples, and *X*_*i*_ is the ith sample. Second, the covariance between sample X and sample Y is calculated, see Eq (3):

$$Cov(X,Y)=E((X-E(X))(Y-E(Y)))=\frac{1}{n-1}\sum (X_{i}-\bar{x})(Y_{i}-\bar{Y})$$ (3)

where E(X) is the expectation of the variable X and $\bar{X}$ is the mean value of the variable X. When Cov(X, Y) is positive, it means that X and Y are positively correlated, when it is negative, it means that X and Y are negatively correlated, and when it is zero, it means that X and Y are independent of each other. Therefore, the formula for calculating covariance can see Eq (4):

$$Cov(X,Y\ldots \ldots Z)=(\begin{array}{llll} Cov(x,x) & Cov(x,y) & \ldots \ldots & Cov(x,z)\\ Cov(y,x) & Cov(y,y) & \ldots \ldots & Cov(y,x)\\ \ldots \ldots & \ldots \ldots & \ldots \ldots & \ldots \ldots \\ Cov(z,x) & Cov(z,y) & \ldots \ldots & Cov(z,z) \end{array})$$ (4)

where Cov(X,Y,……, Z) is the covariance between variables X, Y,……, and Z. The non-diagonal line is the covariance between samples and the variance of the variables on the diagonal.

#### Hash matrix

i.e., the covariance matrix multiplied by (total data volume—1). The eigenvalues and eigenvectors of the matrix are the same, so calculating the new mean and variance can see Eqs (5) and (6):

$$m=\frac{1}{n}\overset{n}{\underset{k=1}{\sum }}X_{k}$$ (5)

$$S=\overset{n}{\underset{k=1}{\sum }}(X_{k}-m){\left(X_{k}-m\right)}^{T}$$ (6)

where m is the new mean, S is the new variance, X_k_ is the kth sample, and n is the number of samples.

#### Eigenvalue decomposition matrix

See Eq (7):

Au=λu (7)

where λ is the eigenvalue corresponding to the eigenvector v, and a set of eigenvectors of a matrix is a set of orthogonal eigenvectors. The eigenvalue decomposition matrix, for matrix A, has a set of eigenvectors v. By orthogonalizing this set of eigenvectors, a set of orthogonal unit vectors can be obtained.

RETRACTED

The eigenvalue decomposition, i.e., see Eq (8), where A is a matrix, Q is the eigenvector matrix of matrix A, ∑ is a diagonal array, and the elements on the diagonal are eigenvalues.

$$A=Q{\Sigma \Sigma }^{-1}$$ (8)

#### SVD decomposition matrix

There is always a singular value decomposition for any matrix A, see Eq (9):

$$A=U\Sigma \Sigma^{T}$$ (9)

where U is the n * n-dimensional matrix formed by the eigenvectors of matrix A, ∑ is the n * n-dimensional diagonal array with n eigenvalues as the dominant diagonal, and UT is the n * n-dimensional transpose matrix formed by the eigenvectors of matrix A. The covariance matrix is based on the eigenvalue decomposition of the covariance matrix.

#### The PCA algorithm is implemented based on the eigenvalue decomposition covariance matrix

i.e., de-averaging (i.e., decentering), subtracting each feature from its average value, and calculating the covariance matrix, see Eq (10):

$$\frac{1}{n}XX^{T}$$ (10)

where X = {X1,X2,…, Xn}is the input data.

The eigenvalues and eigenvectors of the covariance matrix are obtained by eigenvalue decomposition (see Eqs (7) and (8)), and the largest k eigenvalues are selected by sorting the obtained eigenvalues from largest to smallest. Finally, the eigenvector corresponding to the largest k eigenvalues is used as a row vector to form a new eigenvector matrix P. Finally, the data is transformed into the new space constructed by the k eigenvectors, see Eq (11).

Y=PX (11)

Using multiple linear regression equations, see Eq (12):

$$y=\beta_{0}+\beta_{1}x_{1}+\beta_{2}x_{2}+\ldots \ldots +\beta_{k}x_{k}+\varepsilon$$ (12)

where β_0_, β_1_, β_2_,……β_k_ is k+1 unknown parameters, β_0_ is the regression constant, β_0_, β_1_, β_2_,……β_k_ is the regression coefficient, y is the explained variable, general variables X_1_, X_2_,…… X_k_ are k general variables that can be precisely controlled and are called explanatory variables.

Certain assumptions are first made about the multiple linear regression equation, see Eqs (13) and (14):

E(ε)=0 (13)

$$\text{var}(\varepsilon )=\delta^{2}$$ (14)

where ε is the random error, E(ε) is the expectation of the linear regression equation, and var(ε) is the variance of the linear regression equation.

The least squares method is also used to estimate the regression coefficients in the multiple linear regression equation. To determine the degree of goodness of fit of the multiple linear regression, multiple coefficients of determination are used, see Eq (15):

$$R^{2}=\frac{SSR}{SST}=1-\frac{SSE}{SST}=1-\frac{\sum {\left(y-y\right)}^{2}}{\sum {\left(y-\bar{y}\right)}^{2}}$$ (15)

where SSE is the squared sum of residuals, SST is the squared sum of total deviations, and SSR is the squared sum of regressions.

0 ≤ R^2^ ≤ 1. The closer the R^2^ is to 1, the better the regression plane fit, and conversely, the closer the R^2^ is to 0, the lower the fit. In the actual fitting process, as the number of variables increases, the regression squared sum (SSR) increases and so does R^2^. Therefore, when comparing the degree of fit between regression equations applying different numbers of variables, R^2^ must be corrected, see Eq (16):

$${\bar{R}}^{2}=1-\frac{SSE/(n-k-1)}{SST/(n-1)}=1-\frac{SSE}{SST}\cdot \frac{n-1}{n-k-1}=1-(1-R^{2})\frac{n-1}{n-k-1}$$ (16)

where SSE is the squared sum of residuals and SST is the squared sum of total deviations.

RETRACTED

The F statistic is used to measure the fit of the regression equation, and the formula for the F statistic is transformed in combination with the formula for R2, see Eq (17). If the fit of the regression equation is high, the more significant the F-statistic is, and the more significant the F-statistic is, the better the fit of the regression equation is.

$$F=\frac{R^{2}/k}{\left(1-R^{2})/(n-k-1\right)}$$ (17)

### 2. Model building and analysis

Use the SPSS (a mathematical analysis software) to reduce the dimensionality of the given variables into several main variables, and get the analysis results shown in Table 2.

**Table 2:** Principal component analysis checklist.

KMO	Null	
**Bartlett**	Approximation of the cardinal directions	2655.148
	df	15
	p-value	0.000

In Table 2, the p-value of Bartlett’s test is less than 0.05, indicating that the model is suitable for principal component analysis. The null KMO value indicates that the collected data are not very sensitive to principal component analysis, which is one of the shortcomings of the modeling.

A total of two principal components were extracted, and spss was used to derive the variance explained by each principal component and the cumulative total variance explained by each component, as shown in Table 3.

**Table 3:** Explanation of variance.

No.	Feature Root			Main Ingredient Extraction		
	Feature Root	Variance Explanation Ratio %	Cumulative %	Feature Root	Variance Explanation Ratio %	Cumulative %
1	4.327	72.116	72.116	4.327	72.116	72.116
2	0.986	16.431	88.546	0.986	16.431	88.548
3	0.644	10.736	99.282			
4	0.030	0.495	99.778			
5	0.013	0.222	100.000			
6	0.000	0.000	100.000			

The explanatory ratios for the variance of the two principal components were 72.116% and 16.431%, respectively, and the cumulative explanatory ratio was 88.546%. The weighted explanatory ratios, or weights, for the principal components are 72.116/88.546 = 81.44% and 16.431/88.546 = 18.56%, respectively.

RETRACTED

The correspondence between each principal component and the studied data variables can be derived from the values of the loadings in Table 4, where the studied data correspond to a common degree value higher than 0.4, which means that there is a strong correlation between the studied data and the principal components, ensuring that most of the information in the studied data variables can be extracted from the principal components. Finally, weighting was performed using principal component analysis to analyze the correspondence between the principal components and the studied data variables as shown in Table 5.

**Table 4:** Table of principal component load factors.

Variable Name	Load factor		Communaliy (Metric variance)
	Main ingredient 1	Main ingredient 2	
Total Expenditures for Mass Cultural Institutions	0.976	-0.021	0.952
Number of Cultural Centers	-0.630	-0.261	0.465
Total Attendance at Artistic Venues	-0.216	0.956	0.962
Performing Arts Group Performance Revenue	0.983	0.046	0.968
Number of performing arts groups	0.991	0.009	0.983

**Table 5:** Component score coefficient matrix.

Variable Name	Composition	
	Composition 1	Composition 2
Total Expenditures for Mass Cultural Institutions	0.225	-0.021
Number of Cultural Centers	-0.146	-0.265
Total Attendance at Artistic Venues	-0.050	0.970
Performing Arts Group Performance Revenue	0.227	0.047
Number of performing arts groups	0.229	0.009

Component 1 score = 0.225*Total expenditures of mass cultural institutions—0.146*Number of cultural venues—0.050*Total audiences at performing arts venues + 0.227*Performing arts groups + 0.229*Number of performing arts groups + 0.229*Number of performing arts groups.

Component 2 score = -0.021*Total expenditures of mass cultural institutions -0.265*Number of cultural halls +0.970*Total audiences at performing arts venues +0.047*Performing arts groups +0.009*Number of performing arts groups +0.009*Number of performing arts groups.

A linear regression analysis was performed on the two principal components obtained, and the regression analysis was performed using SPSS software to obtain Fig 3, which shows that the two principal component data can be linearly regressed.

**Fig 3:** Scatterplot of principal component variables.

Calculation of the summary of the number of performing arts venues model using the spss software, see Table 6.

**Table 6:** Summary of the number of performing arts venues model.

Model	R	R2	Adjusted R2	Errors in Standard Estimates	Durbin-Watson Index
1	647a	418	321	335.33639	903

Where a refers to predictor variables that have variables 1 and 2, respectively. The range of values for the coefficient a is shown in Table 7.

RETRACTED

**Table 7:** Test and value of the coefficient a.

Model		Unstandardized Coefficients		Standardization Factor	t	Significance	95% confidence interval for B	
		B	Standard Error	Beta			Lower Limit	Upper Limit
1	Constants	1267.124	195.741		6.473	0	840.640	1693.608
	Variable 1	0	0	1.166	2.776	17	0	0
	Variable 2	2	1	783	1.863	87	0	3

Analysis of variance (ANOVA) on the model of the number of performing arts venues using the spss software, as shown in Table 8.

**Table 8:** Analysis of variance.

Model		Sum of Squares	Degree of Freedom	Mean Square	F	Significance
1	Regression	969513.774	2	484756.887	4.311	39b
	Residual	1349405.959	12	112450.497		
	Analysis	2318919.733	14			

Where b is the dependent variable and is the number of performing arts venues.

The regressions on the standardized residuals are shown in Fig 4.

**Fig 4:** Normal P-P plots of regression standardized residuals.

When P < 0.001, it indicates that there is a linear correlation between the dependent variable and the independent variable. If P>0.05, the regression is not statistically significant and there is no linear correlation between the dependent variable and the independent variable. Our P = 0.039<0.05, so there is a linear relationship in the model.

Two principal components (named Component 1 and Component 2, which are different from the existing components and can be characterized by the existing components) are derived from multiple components through principal component analysis and a binary linear regression model is fitted through these two principal components. The normal P-P plot of the regression standardized deviation of the residuals in Fig 4 shows that there is a linear relationship between the two principal components and the performing arts venues, and it conforms to a normal distribution.

## Suggestions and prospects

The protection and inheritance of folk art in the network needs to form a systematic and complete knowledge base in the network. Based on this, we should make breakthroughs in four aspects: talent, content, influence and supervision to promote the development of folk art [8–13].

### 1. Cultivate compound talents for folk art communication through network

Nowadays, culture and tourism develop together, and the tourism industry has created good conditions for the objective materialization of folk art [8], folk artists take advantage of the opportunity of the fusion of culture and tourism to innovate traditional art forms and integrate them with the characteristics and expressions of the new era. However, this requires professionals to escort the whole process of folk art production/in production.

RETRACTED

Therefore, Talents are the necessary driving force to push forward a certain cause. In the network era, folk art protection and inherit can’t leave the help of the network. Our country pays great attention to cyberspace and cyber culture, so it is an important era node to cultivate computer and art composite talents with good knowledge reserve. The first thing we should pay attention to is students’ knowledge learning of art and training their cognition about the prospect of the industry from the whole. In addition, colleges and universities should carry out some relevant comprehensive courses and knowledge lectures, such as computer, network, new media, communication, etc. to increase the competitiveness of students in combination with the needs of enterprises. In addition, the postgraduate examination contents of professional courses should be set scientifically to reflect the candidates’ solid professional knowledge and other necessary professional related knowledge.

The society needs to help the cultivation of talents. The problems of enterprises [14–16] and social organizations in the process of actual operation should be discussed and fed back with colleges and universities in time to promote the curriculum setting. Besides, more extracurricular practical activities should be carried out to give compound talents the opportunity to solve the problems encountered in the field in the cultivation stage by using their own knowledge and foster their abilities to transform knowledge into problem solving.

### 2. Build a cultural brand of folk art network communication

Since high quality is, but the systematic creation of high-quality products can be the key to win the hearts of the public and better promote the development of the cause. Professional service-oriented companies [11,12,17–20] need to sort out the high-quality content from two aspects of market and art content. The classification will help to explore the overall context by using big data analysis technology, which will become an important branch of the Chinese cultural network, and help to present a more professional and systematic form of expression to the public and arouse their interest to a greater extent.

Now, for example, after the first film of Hollywood series becomes popular, the follow-up films will receive continuous attention. Although the series will bring certain visual fatigue, the box office is still high. The systematic art and cultural products have brought the audience into a new world where everything needs to be redefined. Under the guidance of a series of fresh feelings, the public gradually contacts the connotation behind it and add some online and offline activities with ritual to stimulate sustained interest. In the process of combining with film and television, we should accurately grasp the context behind folk art and make it an inexhaustible source, not just give up the real meaning to please the audience, but also select the points that meet the current audience’s cognitive level or the hot spots of the times, such as the garbage classification of spider man, which will cause a boom. After doing this, movies, comics and so on will take this as the background to build a brand chain belonging to folk art.

RETRACTED

Some characteristic activity locations such as theme bars, theme restaurants, etc. where can create an atmosphere of folk art, so as to gather a group of like-minded artists will promote the communication and dialogue of folk artists, Regular informal party activities will be different from formal seminars, symposiums, etc. In a relaxed and familiar environment, a series of activities such as thought collision and brainstorming are carried out. A series of inadvertent details are conducive to the burst of new inspiration and the production of high-quality works. Collaborating with the community, kindergartens, etc. to hold hands-on activities for children during traditional holidays is an option. On the one hand, it can leverage children’s imagination and curiosity to provide fresh blood for the redevelopment of traditional arts; on the other hand, it can increase children’s participation in social activities [9], promote the effective dissemination of traditional arts in the family as a social "cell", and increase visibility and recognition.

Playing game caters to people’s preferences, that is a phenomenon we can’t ignore. It would be a good source of creation for game developers to add some elements of folk art among game background, scene, characters and game plot development, since we have a lot of yearning life scenes in China’s excellent culture.

### 3. Enhance the carrying capacity of cultural heritage of folk art network communication

The spread of folk art through the Internet can improve the communication efficiency, expand the influence, and facilitate the inheritance of folk art. Besides, it can help the masses to open the mysterious door of folk art, promote the masses to understand the traditional culture of the Chinese nation and stimulate and gather the masses’ sense of identity and belonging to their own national culture.

Network literature is an important component of Chinese culture spreading in cyberspace. Behind the network literature is the growing number of users, reaching 432 million in 2018, as shown in Fig 5. Users enter the world outlined by the author through computers, mobile phones, tablets and other carriers, temporarily divorced from the real society, and get spiritual release. In this process, the elements of folk art and culture in literary works will not only improve their interest, but also affect the readers to feel the connotation behind culture to varying degrees through the description of the natural plots and details of literary work.

RETRACTED

**Fig 5:** China’s online literature user scale in 2012–2018 Unit: 100 million people. Source: CNNIC, China Industrial Research Institute.

The inheritors of folk art need to be protected too. They may not have the deep cognitive and creative power of predecessors, but the art they inherit and the endeavor they make is precious. Self media can play their role in helping these inheritors to show their art in the network and expand their influence to the next generation, and finally spread these historical memories. Based on digital technology, a digital art information database is established, and traditional folk art cultural texts are organized into data, which is convenient for future research and learning.

### 4. Build the defense line of folk art network communication

In the process of network communication of folk art, the reasonable communication and feedback between the cultural management department and the public is an important demand to ensure the good development of this cause. In the age of interaction and immediacy [10], the new media platforms such as official micro-blog and WeChat public need to enhance instant communication so as to ensure the effectiveness of platform communication and feedback. Cultural management departments can increase face-to-face communication with folk artists and record the problems existed and adjust the policies accordingly. In this way, we can enhance their trust in cultural management departments, and jointly promote the development of folk art and culture protection and inheritance.

The talent pool, led by the government and composed of experts from various fields such as folk artists, computer network talents and communication scholars, can enter the frontier land acquisition of network supervision from a certain experimental area, train the intelligent supervision system through real cases for the intelligent supervision system, and discuss different situations in the early stage, so as to iterate out the scientific defense system and finally extended to the whole country. The offline talent pool has been transformed into an emergency system to make timely adjustments to the feedback voice from the people.

RETRACTED

## Conclusions

Folk art are rooted in Chinese culture. Behind the protection and inheritance of folk art, it is carried out under the high concern of Chinese traditional culture at the national level. It is related to the cultural confidence of the Chinese nation in local culture and the development of Chinese cultural industry. This cause requires a lot of time, energy and financial resources from the state and society. Through continuous excavation, analysis, innovation and iteration, these traces from the ancient memory will shine brilliantly in the modern society. This is a long process for people to raise the awareness of protection and recognition to a certain height.

From the perspective of network culture governance, the protection and inheritance of folk art need online and offline collaborative efforts. Government departments need to have necessary and effective supervision and policy-making functions. As the backbone of society, enterprises, universities and cultural centers need to play their functions of cultivating talents, grasping market rules, bringing social and economic benefits, and disseminating folk art and culture in order to form a virtuous circle of discovering new problems and promoting technological progress. The Internet users need to cooperate with the government and social organizations to do their best to contribute to this cause while actively improving their comprehensive quality. The inheritors of folk art should dare to use self-Media to make voice and try to innovate. With the joint efforts of various forces, we can realize the multi-win of all parties, inject new blood into folk art and culture, and make it glow with vigorous vitality in the network era.

## Supporting information

S1 Data (RAR)

## References

[1] JiaL. Research on the Spreading Ecology of Folk Art in the New Era. EKOLOJI. 2019;28(107): 3027–3034.

[2] JinpingXi. Speaking at the Symposium on Literature and Art 2014 10 15 [cited 15 October 2014]. In: People’s Daily Online. Beijing: [Internet]. http://culture.people.com.cn/n/2014/1015/c22219-25842812.html.

[3] YanzuLi. Contemporary Folk Art as a Cultural Industry. Art Observation. 2003;12: 79–80.

[4] ZhaodongXia. New Ideas of Folk Art Protection and Communication in the Era of New Media. Beauty and Time (I). 2015;02: 32–33.

[5] AlakaWali. Destination Culture: Tourism, Museums, and Heritage. AM ANTHROPOL. 1999;101(3): 485–703.

[6] JiyingLiu, QingLu. Research on the Protection of Folk Art and Culture from the Perspective of Cultural Governance. Journal of Xi’an University of Technology. 2019;39 (03): 359–366.

RETRACTED

[7] HuilinHu. Cultural Governance in China: the Space of Contemporary Chinese Cultural Policy. Shanghai Culture. 2015;02:5–13+125.

[8] HashimotoH. Between preservation and tourism: Folk performing arts in contemporary Japan. Asian Folklore Stud. 2003;62(2): 225–236.

[9] Glaveanu, PetreV. Creativity development in community contexts: The case of folk art. Think Skills Creat. 2013;9:152–164.

[10] XingdongFang, JingZhang and XiaorongZhang. Communication mechanism and network governance in real-time network era.Modern communication (journal of communication university of China). 2011;05:64–69.

[11] AndreaCaputo, Ayoko OluremiB. and AmooNii. The moderating role of cultural intelligence in the relationship between cultural orientations and conflict management styles. J Bus Res. 2018;89: 10–20.

[12] ZhiChen, ShenglanHuang, ChongLiu and et al Fit between Organizational Culture and Innovation Strategy: Implications for Innovation Performance. SUSTAINABILITY. 2018;10(10): 3378.

[13] VictoriaEugenia Garcia-Vera; AntonioJose Tenza-Abril; MarcosLanzon; et al Exposing Sustainable Mortars with Nanosilica, Zinc Stearate, and Ethyl Silicate Coating to Sulfuric Acid Attack. SUSTAINABILITY. 2018;10(10): 3769.

[14] AliAlkhuraiji; ShaofengLiu; Festus OluseyiOderanti; et al New structured knowledge network for strategic decision-making in IT innovative and implementable projects. J Bus Res. 2016;69(5): 1534–1538.

[15] PeymanAkhavan, MahdiHosseini S. Social capital, knowledge sharing, and innovation capability: an empirical study of R&D teams in Iran. TECHNOL ANAL STRATEG. 2016;28(1): 96–113.

[16] MuradAli, KonanKan SenyAnderson and MarkoSarstedt. Direct and configurational paths of absorptive capacity and organizational innovation to successful organizational performance. J Bus Res. 2016;69(11): Pages: 5317–5323.

[17] MajidDarroudi; MaryamBagherpour; Hasan AliHosseini; et al Biopolymer-assisted green synthesis and characterization of calcium hydroxide nanoparticles. CERAM INT. 2016;42(3): 3816–3819.

[18] Nagy-SándorZsuzsa, BerkersP. Culture, Heritage, Art: Navigating Authenticities in Contemporary Hungarian Folk Singing. CULT SOCIOL. 2018; 12(3). 10.1177/1749975518780770 30369961PMC6187076

[19] BronnerSimon J. Investigating Identity and Expression in Folk Art. Winterthur. 1981;16(1): 65–83.

[20] ToelkenBarre. The Heritage Arts Imperative. JAF. 2003116(460): 196–205.

